# Influences of miR-378a-3p on the Pathogenesis of Allergic Rhinitis via GzmB-Mediated Inflammatory Reaction

**DOI:** 10.1155/2022/5926834

**Published:** 2022-08-29

**Authors:** Xuping Wang, Haiqing Zhang, Long Du, Lian Zhang

**Affiliations:** Department of ENT, Affiliated Taikang Xianlin Drum Tower Hospital, Medical School of Nanjing University, Nanjing, Jiangsu 210000, China

## Abstract

**Methods:**

Totally, 24 BALB/c mice were assigned to the AR group, control group, GzmB group, and blank group (each *n* = 6). The blank group was normally fed without treatment, and the other three groups were treated by ovalbumin (OVA) to induce AR models, in which the GzmB group was intranasally injected with lentiviral vector suppressing GzmB expression during the second immunization, while the control group was given the GzmB-blank vector. The times of AR pathological behaviours such as sneezing and scratching the nose of mice were observed and counted. The nasal lavage fluid of each mouse was acquired, and then, the mouse was executed by cervical dislocation, followed by collection of blood and nasal mucosa tissues. Then, ELISA was adopted for quantifying immunoglobulin E (IgE), interleukin (IL)-4, IL-6, and histamine (HA), and nasal mucosa tissues were treated by HE and TUNEL staining to observing their histopathological manifestations. PCR and western blot (WB) were adopted for quantifying GzmB and miR-378a-3p. Additionally, with NP69 cells, dual luciferase reporter (DLR) assay was carried out for determining the targeting association of GzmB with miR-378a-3p. Another 24 mice were assigned to the AR group, GzmB group, miR-378a-3p group, and GzmB+ miR-378a-3p group (each *n* = 6). The AR and GzmB groups were treated as above. The miR-378a-3p group was intervened by lentiviral vector suppressing miR-378a-3p, while the GzmB+ miR-378a-3p group was given GzmB and lentiviral vector suppressing miR-378a-3p meantime. A rescue assay was conducted through repeating the above tests.

**Results:**

The times of sneezing and rubbing the nose and the levels of IgE, IL-4, IL-6, and HA were similar between the control and AR groups (all *P* > 0.05), and these items of the two groups were all higher than those of the blank and GzmB groups (all *P* < 0.05). However, no notable difference was observed in IL-4 and IL-6 levels between the GzmB and blank groups (both *P* > 0.05), while higher levels of other detection results were found in the former group than in the latter (all *P* < 0.05). The staining results revealed obvious congestion, oedema, and necrosis structures in the nasal mucosa epithelium of the control and AR groups and also revealed a large number of infiltrating eosinophils and notable increase of apoptotic nasal mucosa epithelial cells. The GzmB group showed notably improved nasal mucosa tissues, and its infiltration and apoptosis of eosinophils were more notable than those of the blank group, but notably weaker than those of the AR and control groups. Additionally, the PCR and WB results revealed similar miR-378a-3p and GzmB levels in nasal mucosa between the control and AR groups (both *P* > 0.05), and a notable decrease of miR-378a-3p and a notable increase of GzmB in both groups (both *P* < 0.05). The DLR **a**ssay revealed notably suppressed fluorescence activity of GzmB-WT in NP69 cells after transfection of miR-378a-3p mimics (*P* < 0.05) and notably down regulated GzmB protein after increase of miR-378a-3p (*P*<0.05). Finally, the rescue assay revealed that downregulating miR-378a-3p aggravated the pathological changes of AR (*P* < 0.05) and also completely reversed the impacts of inhibiting GzmB on the pathological behaviours of AR mice.

**Conclusions:**

MiR-378a-3p can accelerate the pathological development of AR through targeted inhibition on the release of pro-inflammatory factors such as IgE and HA activated by GzmB, so it is a promising molecular target of AR therapy and offers a novel research direction for the complete cure of AR.

## 1. Introduction

Allergic rhinitis (AR), primarily mediated by immunoglobulin E (IgE), is a noninfectious inflammatory disease of nasal mucosa [1]. As a frequently seen chronic inflammation of the upper respiratory tract, AR presents a growing incidence worldwide [2]. According to the surgery, over 500 million patients suffer AR worldwide and the incidence even reaches approximate 12–30% in some developed countries [3]. Allergens such as inhalant substance and food can trigger AR, and the manifestations and severity of different types of AR are inconsistent. At the current stage, there lacks complete cure scheme for it in clinical practice, and the treatment principle is still to avoid allergens as much as possible [4]. AR is one primary pathogenic factor of asthma, and it can even trigger acute respiratory dysfunction and failure and endanger life safety in severe cases [5]. Most pathological conditions of AR can be effectively controlled, but over 50,000–80,000 patients die from AR every year worldwide [6], so clinical researchers and patients must focus on the prevention and therapy of AR.

Over the past few years, as research deepens, AR is clinically found to be a multifactorial inflammatory disease triggered by the interaction of genes and environment, and its various phenotypes are under strong genetic control [7]. At the current stage, reportedly, many genes and associated transcription factors are implicated in the pathogenesis of AR by regulating inflammatory reaction. For example, Li et al. [8] have indicated the participation of differentiated Th9 cells that were activated by IRF4 transcription in AR, and Zhang et al. [9] have indicated the positive influences of NLRP3 inhibitor on the pathological development of AR. The modern research on the pro-inflammatory mechanism molecularly offers a new direction for the early therapy AR in the future and also reveals the potential therapeutic targets of AR, which is known as the breakthrough of diagnosis and therapy of AR [10]. Accordingly, this study screened the potential genes with aberrant expression through the GSE43523 data set in GEO and found granzyme B (GzmB) among them. Prior research on GzmB primarily focused on the impacts of GzmB on tumour diseases [11, 12], but did not point out its potential association with AR. However, Tschopp et al. [13] have clearly pointed out GzmB as a novel allergic inflammatory mediator able to induce blood basophils and release in large quantities in asthma cases. Accordingly, we suspect that there exist possible influences of GzmB on the occurrence of AR, but no research has yet confirmed this view. As everyone knows, the activation state of transcription factors is often regulated by microRNA (miRNA), and the function of multiple miRNAs in AR has also been repeatedly confirmed clinically [14]. Thus, we analysed miRNAs that were possibly targeted by GzmB through the online target gene forecasting website and found miR-378a-3p among the miRNA family strongly associated with the process of cellular inflammatory response [15]. Caserta et al. [16] have pointed out that miR-378a-3p is one miRNA strongly bound up with the severity of systemic inflammatory response syndrome.

In the face of the increasing incidence of AR, it is of great reference value to determine the pathogenic mechanism of AR molecularly for ensuring the safety of patients and curing AR in the future. Accordingly, this study analysed the impacts of miR-378a-3p and GzmB on AR to set the foundation for the follow-up associated research and offer novel ideas and directions for the future diagnosis and therapy of AR.

## 2. Materials and Methods

### 2.1. Bioinformatics Analysis

We the keyword “allergic rhinitis” to search for relevant information from the GEO (https://www.ncbi.nlm.nih.gov/geo/) with the first choice of organisms in the screening results as “homo sapiens,” and then reviewed the results one by one. Finally, “global gene expression in nasal epithelial cells of patients with seasonal allergic rhinitis” was selected as the research object, and the public dataset GSE43523, including 12 sets of samples (5 groups of nonallergic control subjects and 7 groups of seasonal AR patients), was obtained for analysis. Based on TargetScan (https://www.targetscan.org/vert_72/), miRDB (https://mirdb.org/mirdb/index.html), and miRWalk (https://mirwalk.umm.uni-heidelberg.de/), the potential target upstream miRNAs of GzmB were searched and all put into the Wayne diagram matrix. Finally, the target genes co-existing in the above three platforms were used as the potential target genes of GzmB, and the complementary binding loci were obtained.

### 2.2. Data of Animals

Totally, 48 BALB/c mice offered by Beijing Animal Science Co., Ltd. (animal experimentation license: SYXK (Beijing) 2020–0050) were caged (3 mice/cage) and kept in a biological hazard containment facility without specific pathogens in a 12-hour day/night cycle (20 ± 1°C) and with free access to food and water. Totally, 24 mice were chosen in a random manner and assigned to the AR group, control group, GzmB group, and blank group (each *n* = 6).

### 2.3. Constructions of Animal Models

The blank group was not treated, and other groups were treated to establish AR models based on the research of Van Nguyen et al. [17] after 1-week adaptive feeding. Specifically, normal saline (200 *μ*L) with 25 *μ*g ovalbumin (OVA) and 2 mg aluminium hydroxide was injected intraperitoneally into the mouse on the 10^th^, 7^th^, and 14^th^ day to promote primary sensitization. One week after sensitization, the second immunization was established. Normal saline (20 *μ*L) diluted with 3% OVA was adopted for attacking mice intranasally every day from 21 d to 35 d. Every mouse in the GzmB group was injected intranasally with lentiviral vector (1 × 10^7^ IFUs) inhibiting GzmB expression 3 h before the second immunization from 28 d to 34 d. Mice in the control group were injected intranasally with GzmB-blank lentiviral vector (1 × 10^7^ IFUs) after secondary immunization from 28 d to 34 d. The lentiviral vector was constructed and designed by GenScript Biotechnology Co., Ltd.

### 2.4. Mouse Behaviour Analysis and Sample Collection

At 35 days after modelling, the times of sneezing and rubbing the nose of mice in each group within 10 minutes were recorded. Then, the mice were anaesthetized by intraperitoneal injection of pentobarbital sodium (50 mg/kg), and them executed by cervical dislocation, followed by separation of the trachea and inserting of the catheter into the nasopharynx. Precooled PBS (1 ml) was injected into the catheter and was let to flow out through bilateral anterior nostril, and nasal lavage fluid was collected 3 times. Subsequently, the nasal mucosa tissues and blood specimens of mice were acquired for subsequent detection.

### 2.5. ELISA

Nasal lavage fluid, as well as blood that was placed in coagulation tubes and left standing at room temperature for 30 min, were centrifuged (1505 × *g*, 4°C) for 10 min to obtain the supernatant and serum. Lavage fluid and serum IgE, interleukin (IL)-4, IL-6, and histamine (HA) were examined under the instructions of ELISA kits.

### 2.6. Histological Observation

The nasal mucosa tissues of mice were conventionally embedded in paraffin and sectioned, and then placed in a temperature box at 60°C for 2 h, followed by drying and sectioning. After that, the sections were dewaxed with xylene, dehydrated with gradient ethanol, and soaked successively with haematoxylin and eosin for 5 min and 3 min, respectively. The histopathological changes were observed under a microscope after routine dehydration, transparency, drying, and mounting.

### 2.7. TUNEL Staining

The nasal mucosa tissues of mice were trypsinized for 30 min, followed by washing via PBS and 1-h incubation with low-priced labelling solution and transforming agent. Subsequently, NBT/BCIP was adopted for colour development, followed by gradient ethanol dehydration. Then, the tissues were made to be transparent in xylene, followed by sealing with neutral gum. The positive cells were counted under fluorescence microscope (×20), on which the number of apoptotic cells/50 *μ*m nasal mucosa epithelial tissues was calculated.

### 2.8. qRT-PCR Assay

Total RNA acquired from nasal mucosa tissues by TRIzol was determined by an ultraviolet spectrophotometer to understand its purity. Total RNA (5 *μ*g) was treated by reverse transcription under the guidelines of a RT Primer kit to acquire cDNA, and then, the primers, SYBR Green, and 2xTaq PCR Master Mix were adopted for qRT-PCR conditions: 95°C for 5 min, 95°C for 10 s, 60°C for 30 s, and a total of 40 cycles. GenScript USA Inc (Nanjing) designed and constructed all the primer sequences of this study (Table 1), and 2^−△△CT^ was adopted for relative expression calculation.

### 2.9. Western Blot (WB) Assay

RIPA lysis buffer was adopted for extracting total protein from nasal mucosa. After purity determination of the total protein by BCA, 10–20 *μ*g was treated by SDS-PAGE, followed by transfer to a PVDF. The membrane was treated by 1-h immersion (room temperature) in 5% defatted milk, followed by the addition of GzmB (1 : 1000) and GAPDH (1 : 1000) type I antibody and overnight incubation (4°C). Then, the membrane was treated by cleaning via TBST, followed by 1-h incubation with type II antibody (1 : 2000). Subsequently, ECL was adopted for development, and Image*J* was adopted for analysing the target grey value.

### 2.10. Dual Luciferase Reporter (DLR) Assay

NP69 cells were offered by ATCC. Log-phase NP69 cells were placed in a 12-well plate. After their confluency reached 70–80%, wild-type (WT) and mutant (MUT) GzmB 3′-UTR were cloned into pmirGLO plasmid, and the miR-378a-3p mimic sequence (miR-378a-3p mimics) and negative control sequence (miR-378a-3p-NC) were co-transfected into NP69 cells, Finally, the fluorescence activity was detected under the instructions of a luciferase detection kit.

### 2.11. Rescue Assay

The remaining 24 mice were assigned to the AR group, GzmB group, miR-378a-3p group, and GzmB+ miR-378a-3p group in a random manner (each *n* = 6). The AR and GzmB groups were treated as above. The miR-378a-3p group was intervened by lentiviral vector suppressing miR-378a-3p 3 h before the second immunization from 28 days to 34 days. The GzmB+ miR-378a-3p group was injected with GzmB and lentiviral vector suppressing miR-378a-3p meantime. The sneezing and scratching behaviours of mice were recorded according to the above methods, and the nasal lavage fluid and nasal mucosa tissue samples were acquired for the quantification of IgE, IL-4, IL-6, HA, and pathological conditions of nasal mucosa.

### 2.12. Statistical Analyses

This study adopted SPSS22.0 for statistical analyses and GraphPad for graphic drawing. All the results were presented by the $\bar{\chi }\pm s$, and multigroup comparison was conducted using the repeated measures ANOVA and post hoc LSD test. *P* < 0.05 suggests a notable difference.

## 3. Results

### 3.1. Bioinformatics Analysis Results

Firstly, genes with differential expression in AR cases were screened through the GEO, and such genes in nonallergic control subjects and AR patients were analysed through GEOR2. The results were screened with Log (FC) > 1 or <−1 and *P* < 0.05, and corresponding volcano map and heat map were plotted. Then, PPI network was analysed via the STRING database (https://string-db.org/) to understand the associations among different genes. Then, through GO enrichment analysis according to the expression of differential genes, genes with the most notable difference were obtained, including GzmB as seen in Figure 1.

### 3.2. Comparison between Behaviours and Pathological Changes of AR in Mice

No mouse developed peritonitis in the experiment, and one mouse in the control group died, presumably due to asphyxia. The results of mouse behaviour test revealed no difference between the control and AR groups in the times of sneezing and rubbing the nose (*P* > 0.05), more times of them in the control and AR groups than in the blank and GzmB groups (*P* < 0.05), and more times of them in the GzmB group than in the blank group (*P* < 0.05). The ELISA results revealed no notable differences between the control and AR groups in IgE, IL-4, IL-6, and HA levels in nasal lavage fluid and serum (all *P* > 0.05) and higher levels of them in the control and AR groups than in the blank and GzmB groups (all *P* < 0.05). Moreover, the GzmB group presented higher IgE and HA levels than the blank group and showed no difference with the blank group in IL-4 and IL-6 levels (both *P* < 0.05) as seen in Figure 2.

### 3.3. Comparison of Inflammatory Infiltration of Nasal Mucosa Tissues in Mice

The staining results of nasal mucosa tissues revealed obvious congestion, oedema, and necrosis structures in the nasal mucosa epithelium of the control and AR groups. In addition, there was disordered arrangement of epithelial cells in the nasal mucosa, thinning of the epithelium, loose connection between epithelial cells, and subepithelial and stromal oedema, as well as infiltration of inflammatory cells dominated by a large number of eosinophils. According to the results, in the blank group, the nasal mucosa epithelium was intact and normal, and eosinophils were rare. The GzmB group showed notably improved nasal mucosa tissues, and its infiltration and apoptosis of eosinophils were more notable than those of the blank group, but notably weaker than those of the AR and control groups as seen in Figure 3.

### 3.4. Comparison of Apoptosis of Nasal Mucosa Cells

According to the TUNEL staining results, no notable difference was observed between the control and AR groups in the apoptosis of nasal mucosa cells (*P* > 0.05), but the two groups showed notably increased apoptotic cells in contrast to the GzmB and blank groups (all *P* < 0.05), and the GzmB group showed slightly increased apoptotic cells in nasal mucosa (*P* < 0.05) as seen in Figure 4.

### 3.5. GzmB and miR-378a-3p in AR Cases

According to the detection results, the control and AR groups were similar in the expression of miR-378a-3p and GzmB mRNA in nasal mucosa tissues (both *P* > 0.05), and they showed lower miR-378a-3p expression and higher GzmB mRNA expression than the blank and GzmB groups (both *P* < 0.05). Additionally, the GzmB group showed lower miR-378a-3p expression and higher GzmB mRNA expression than the blank group (both *P* < 0.05). According to the WB assay, the control and AR groups were similar in GzmB protein level (*P* < 0.05), and their GzmB protein level was higher than that in the GzmB and control groups (both *P* < 0.05), with higher level in the GzmB group than in the blank group (*P* < 0.05) as seen in Figure 5.

### 3.6. Verification of the Targeted Association of miR-378a-3p with GzmB

Based on online target gene forecasting website, the targeting association of miR-378a-3p with GzmB was screened, and miR-378a-3p was found to be contained in upstream target genes of GzmB according to TargetScan, miRDB, and miRWalk. The DLR assay revealed notably suppressed fluorescence activity of GzmB-WT after transfection of miR-378a-3p mimics (*P* < 0.05), which verified the targeted regulation of miR-378a-3p to GzmB. The WB revealed notably lower GzmB protein expression in NP69 cells transfected with miR-378a-3p mimics than in those with miR-378a-3p-NC (*P* < 0.05) as seen in Figure 6.

### 3.7. Rescue Assay

No mice developed peritonitis in the experiment, and all the mice were successfully modelled. According to the observation results of mouse behaviours, the times of sneezing and rubbing the nose of the miR-378a-3p + GzmB and AR groups were similar (*P* > 0.05), but higher than those of the GzmB group and lower than those of the miR-378a-3p group (all *P* < 0.05). According to ELISA results, the levels of IgE, IL-4, IL-6, and HA in the miR-378a-3p+ GzmB and AR groups were similar (all *P* > 0.05), but higher than those in the GzmB group and lower than those in the miR-378a-3p group (all *P* < 0.05). The results of HE staining also revealed obvious congestion, oedema, necrosis, and eosinophil infiltration in the miR-378a-3p+ GzmB group, and more severe pathological damage in the miR-378a-3p+ GzmB group than in the GzmB group. Additionally, in contrast to the miR-378a-3p+ GzmB and AR groups, the miR-378a-3p group showed more serious injury and necrosis of nasal mucosa and also showed a large number of infiltrating eosinophils as seen in Figure 7.

## 4. Discussion

As a chronic inflammatory disease involving the activation of various immune cells and the release of cytokines, AR presents a growing incidence over the past few years [18]. Reportedly, when the upper respiratory tract is exposed to allergens, antigen-presenting cells present allergens to Th2 lymphocytes and then induce B cells to differentiate into plasma cells and produce IgE antibodies [19]. Antigen-specific IgE binds to high-affinity IgE receptors on mast cells and basophils and secretes various pro-inflammatory cytokines and chemokines, resulting in inflammatory anaphylaxis [20]. Accordingly, confirming the specific mechanism of small molecule genes in the process of inflammatory allergic reaction is the key to overcome AR clinically. Our study has discovered the aberrant expression of GzmB in GSE43523 dataset and verified the impacts of miR-378a-3p and GzmB in AR for the first time through assays, which is of great reference value for the follow-up research of AR.

In our study, AR mouse models were induced and established by OVA, and their behaviours and pathology were detected. Prior research has also often adopted the above indicators for observation of the pathological development of AR [21, 22]. Similar to prior research [23, 24], the times of sneezing and rubbing the nose, IgE, IL-4, IL-6, and HA levels in the AR group all greatly increased in our study, which can also verify the success of modelling. As everyone knows, IgE is a crucial factor that mediates allergic inflammatory diseases of the respiratory tract, which is primarily produced by plasma cells in the mucosa lamina propria of the respiratory tract and digestive tract [25]. In the pathogenic process of AR, it is the allergen that stimulates respiratory cells, which triggers the generation of a large number of IgE and activates the release of downstream pro-inflammatory factors like IL-4 and IL-6 [26]. HA, an organic nitrogen-containing compound produced by histidine under the action of decarboxylase, can release in large quantities in the case of tissue damage or inflammation and allergic reactions of tissues to relieve blood vessels and increase the wall permeability of capillaries and venules, causing plasma to leak into tissues and triggering local tissue oedema [27]. Taylor-Clark et al. [28] have pointed out the inhibitory role of HA in inflammatory reaction in the pathological process of AR. In the GzmB group, the times of sneezing and rubbing the nose, and IgE, IL-4, IL-6, and HA levels decreased notably, but the IL-4 and IL-6 levels were not greatly different from those in the blank group, which suggested that downregulating GZMB could improve the pathological process of AR. In addition, observation of the pathological damage of nasal mucosa tissues in each group also revealed severely necrotic, congested, and oedematous accompanied by a large number of infiltrating eosinophils in the AR group, which were in agreement with the observation results of nasal mucosa tissues of AR groups [29]. In addition, in the GzmB group, the damage of nasal mucosa tissues was substantially alleviated, and the infiltration of acid granulocytes was notably reduced, which fully indicated the ability of GzmB to alleviate AR and its potential to be a target of AR treatment with the mechanism possibly bound up with the inhibition of the activation of IgE and HA. Moreover, the TUNEL staining results revealed notably weakened apoptosis of nasal mucosa epithelial cells in the GzmB group, suggesting the impacts of suppressing GzmB on improving the apoptosis of nasal mucosa cells. The impacts of GzmB on the cell life cycle have been frequently studied. For instance, GzmB can mediate the apoptosis of enterovirus 71 [30] and accelerate the apoptosis of toxic lymphocytes via the interaction of p53 and Bcl-2 [31]. As for AR, the accelerated apoptosis of normal nasal mucosa epithelial cells directly impacts the normal operation of nasal cavity, which triggers pathological conditions such as nasal congestion and respiratory failure [32]. The impacts of GzmB on nasal mucosa cells once again emphasize its therapeutic potential for AR in the future.

Through the above research, we can preliminarily determine the influence of GzmB on AR, but as we mentioned above, the impact of GzmB may be directly influenced by upstream target, miRNA. As everyone knows, miRNA takes a crucial part in many biological processes like differentiation, migration, apoptosis, and transformation, which primarily induces translation inhibition or post-transcriptional degradation of target gene, mRNA, by binding to 3′UTR of mRNA. Accordingly, for the purpose of determining the upstream regulatory mechanism of GzmB, we screened possible upstream targets, miRNAs, of GzmB through online database and preliminarily judged miR-378a-3p as a possible crucial factor in AR. The follow-up assays revealed a notably increase of GzmB level in AR mice and a decrease of miR-378a-3p level in them, indicating the involvement of GzmB and miR-378a-3p in the development of AR. The increase of miR-378a-3p in the GzmB group also preliminarily revealed the expression association of GzmB with miR-378a-3p. Moreover, the DLR assay in our study revealed notably suppressed fluorescence activity of GzmB-WT in NP69 cells under miR-378a-3p mimics, which indicated a targeted regulation association between them. Finally, the rescue assay revealed that downregulating miR-378a-3p aggravated the pathological changes of AR, and also completely reversed the impacts of inhibiting GzmB on the pathological behaviours of AR mice. Based on the results of the above experiments, we can confirm that miR-378a-3p promotes the inflammatory infiltration of nasal mucosal tissues and accelerates tissue lesions and necrosis through targeted inhibition of GzmB, thus contributing to the development of AR, which also provides more precise guidance for molecular targeted therapy of AR in the future.

However, our study still has many limitations. For example, this study is mainly based on mouse model, but the expression and exact mechanism of miR-378a-3p and GzmB in AR human samples need further confirmation, and the influences of miR-378a-3p targeting AGER on the downstream signal pathway of AR should also be focus of our future research. In addition, we need to do more basic assays *in vitro* to understand more clearly the mechanism of the impacts of miR-378a-3p/AGER on the pathological process of AR, and to conduct more in-depth research and analysis on molecular targeted therapy from the perspective of miR-378a-3p/AGER.

## 5. Conclusion

To sum up, miR-378a-3p can accelerate the pathological development of AR through targeted inhibition on the release of pro-inflammatory factors such as IgE and HA activated by GzmB, so it is a promising molecular target of AR therapy and offers a novel research direction for the complete cure of AR.

## Figures and Tables

**Figure 1:** Bioinformatics analysis results: (a) volcano map of gene expression in GSE43523 data set; (b) volcano map of expression of differential genes; (c) PPI network of expression of differential genes; (d) analysis of the genes with the most notable differences according to enrichment.

**Figure 2:** Comparison between behaviours and pathological changes of AR in mice: (a) comparison of the times of sneezing of mice; (b) comparison of times of rubbing the nose of mice; (c) comparison of IgE level in mouse nasal lavage fluid; (d) comparison of IL-4 level in mouse nasal lavage fluid; (e) comparison of IL-6 level in mouse nasal lavage fluid; (f) comparison of HA level in mouse nasal lavage fluid; (g) comparison of IgE level in mouse serum; (h) comparison of IL-4 level in mouse serum; (i) comparison of IL-6 level in mouse serum; (j) comparison of HA level in mouse serum. ^*∗*^ indicates that there is a difference compared with the blank group (^*∗*^*P* < 0.05). ^#^ indicates that there is a difference compared with the AR group (^#^*P* < 0.05). ^&^ indicates that there is a difference compared with the control group (^&^*P* < 0.05).

**Figure 3:** HE staining results of nasal mucosa tissues.

**Figure 4:** Comparison of apoptosis of nasal mucosa cells: (a) TUNEL staining results; (b) apoptosis of nasal mucosa cells of mice. ^*∗*^ indicates that there is a difference compared with the blank group (^*∗*^*P* < 0.05). ^#^ indicates that there is a difference compared with the AR group (^#^*P* < 0.05). ^&^ indicates that there is a difference compared with the control group (^&^*P* < 0.05).

**Figure 5:** miR-378a-3p and GzmB expression in AR: (a) MiR-378a-3p expression in nasal mucosa tissues of mice; (b) GzmB mRNA expression in nasal mucosa tissues of mice; (c) WB profile; (d) GzmB protein expression in nasal mucosa tissues of mice. ^*∗*^ indicates that there is a difference compared with the blank group (^*∗*^*P* < 0.05). ^#^ indicates that there is a difference compared with the AR group (^#^*P* < 0.05). ^&^ indicates that there is a difference compared with the control group (^&^*P* < 0.05).

**Figure 6:** Verification of the targeted association of miR-378a-3p with GzmB: (a) Wayne diagram of predication of targeted association of miR-378a-3p with GzmB based on online database; (b) complementary binding loci of miR-378a-3p with GzmB; (c) results of DLR assay; (d) western blot image; (e) impacts of miR-378a-3p on GzmB expression in NP69 cells. ^*∗*^ indicates that there is a statistical difference between groups (^*∗*^*P* < 0.05).

**Figure 7:** Rescue assay: (a) comparison of the times of sneezing of mice; (b) comparison of the times of rubbing the nose of mice; (c) comparison of IgE level in mouse nasal lavage fluid; (d) comparison of IL-4 level in mouse nasal lavage fluid; (e) comparison of IL-6 level in mouse nasal lavage fluid; (f) comparison of HA level in mouse nasal lavage fluid; (g) HE staining results of nasal mucosa tissues. ^*∗*^ indicates that there is a difference compared with the AR group (^*∗*^*P* < 0.05). ^#^ indicates that there is a difference compared with the GzmB group (^#^*P* < 0.05). ^&^ indicates that there is a difference compared with the miR-378a-3p group (^&^*P* < 0.05).

**Table 1:** Primer sequences.

	*F* (3′–5′)	*R* (3′–5′)
miR-378a-3p	TCAACTGGTGTC-GTGGAGT	GGGACTGGACTTGGAGTC
U6	GCTTCGGCAGCA-CATATACTAAAAT	CGCTTCAC-GAATTTGCGTGTCAT
GzmB	AGCCTGCACCAAAGTCTCAA	TTTCATTACAGCGGGGGCTT
GAPDH	ACCCACTCCTCCACCTTTGAC	TGTTGCTGTAGCCAAATTCGTT

## Data Availability

The data used to support the findings of the study can be obtained from the corresponding author upon reasonable request.
